# Pathophysiology of aged lymphatic vessels

**DOI:** 10.18632/aging.102213

**Published:** 2019-08-28

**Authors:** Tongyao Shang, Jiangjiu Liang, Carolyn M. Kapron, Ju Liu

**Affiliations:** 1 Medical Research Center, Shandong Provincial Qianfoshan Hospital, Shandong University, Jinan, Shandong, China; 2 Department of Health Care, Shandong Provincial Qianfoshan Hospital, The First Hospital Affiliated with Shandong First Medical University, Jinan, Shandong, China; 3 Department of Biology, Trent University, Peterborough, ON, Canada; 4 Laboratory of Microvascular Medicine, Medical Research Center, Shandong Provincial Qianfoshan Hospital, The First Hospital Affiliated with Shandong First Medical University, Jinan, Shandong, China

**Keywords:** aging, lymphatic vessels, endothelial cells

## Abstract

Lymphatic vessels maintain body homeostasis by recirculation of fluid and cells. Cell senescence induces lymphatic dysfunction. Impaired contractile function is caused by low muscle cell investiture and decrease of nitric oxide in aged lymphatic collectors, leading to poor drainage of lymph. Aging-induced loss of endothelial glycocalyx and production of inflammatory cytokines increases permeability of lymphatic vessels. In addition, aging-associated basal activation of mast cells delays immune response. In this review, we summarize the structural and pathological changes of aged lymphatic vessels, and discuss the underlying molecular mechanisms.

## INTRODUCTION

The lymphatic vascular system functions to regulate tissue fluid transport and facilitate macromolecular absorption [1]. Tissue fluid is collected from the interstitial space by lymphatic capillaries and then transported through collector lymphatic vessels back into the blood stream [1, 2]. The recirculation of fluid and cells through extensive lymph transport is required for the maintenance of homeostasis [3, 4]. Lymphatic vessels are also key routes for the trafficking of immune cells from tissues to lymph nodes during immune responses [5].

The aging process induces changes in structure and function of lymphatic networks [6]. Lymphatic-related diseases are prevalent in elderly, such as lymphedema [7]. In 1960s, the specific “varicose bulges” in muscular lymphatic vessels was observed and this bulges were increased with age [8, 9]. Muscle cell atrophy, elastic elements destruction, and aneurysm-like formations were also found in aged lymphatic vessels [10–12]. Aging associated alterations in lymphatic contractility decrease pump efficiency which result in excessive retention of tissue fluid within interstitial spaces [13, 14]. Reduced responsiveness to inflammatory stimuli in aged lymphatic vessels decreases the normal capacity to react against foreign organisms [15]. The occurrence of high permeability is caused by the loss of glycocalyx and the dysfunction of junctional proteins [6, 16, 17]. In addition, increased caspase-3 activity, the dissociation of the VE-cadherin/catenin complex and the low expression of actin cytoskeleton that occur in aged blood vessels may also be seen in aged lymphatic vessels [16, 18]. Knowledge of the regulatory mechanisms underlying in these disorders is critical to our understanding of the aging-related diseases of lymphatic vessels.

## Structure of lymphatic vessels and their functions in lymph transport

The initial lymphatic vessels are dispersed in the interstitial space of parenchymal organs [6, 19]. These lymphatic capillaries are composed solely of a layer of lymphatic endothelial cells that are directly anchored to the extracellular matrix through filaments [2, 20–22]. The distinctive oak leaf-shaped endothelial cells of initial lymphatics are loosely apposed with overlapping borders and linked with each other by discontinuous, button-like junctions [4, 23]. Regions between buttons are open to allow the entry of fluid and cells without repetitive formation and dissolution of intercellular junctions [4]. These specific structures may function as lymphatic primary valves that prevent the tissue fluid taken up by lymphatic capillaries to be released back into the interstitial space [24] (Figure 1B).

**Figure 1:** **Lymph transport along lymphatic vessels.** (**A**) Unidirectional lymph flow route: lymphatic capillaries collect peripheral tissue fluid and converge into larger collecting vessels, then lymph drains into the lymph node from the afferent lymphatic vessels and flows out from the efferent lymphatic vessel. Afterwards lymph fluid flows through the thoracic duct and the right lymphatic trunk, eventually enters into venous circulation. Arrows indicate the direction of lymph flow. (**B**) Interstitial fluid, macromolecules and immune cells which extravasate from blood vessels are collected by lymphatic capillaries. Initial lymphatics are composed of a layer of oak leaf-shaped endothelial cells and lack of muscle layers. (**C**) Lymphatic collectors contain intraluminal valve and SMC layers that enable the unidirectional lymph flow.

Blind-ended lymphatic capillaries converge into the larger collecting lymphatic vessels [4, 25]. Lymphatic collectors are comprised of spindle-shaped endothelial cells with a complete basement membrane covered by one or more muscle layers [4, 25] (Figure 1C). The secondary valve structures inside the collecting lymphatic vessels separate two adjacent lymphangions to prevent the back-flow of lymph and to overcome opposing pressure gradients [26–28]. Collecting lymphatic endothelial cells are connected to each other through continuous zipper-like junctions, similar to those in blood vessels [4]. The transition from the button-like junctions of initial lymphatics to zippers in collecting lymphatics is typically abrupt in individual vessels [4].

The constituents of lymph include extravasated fluid, macromolecules and immune cells [2]. These elements in peripheral tissues enter initial lymphatic vessels through the opening of primary valves or the vesicular transport of endothelial cells [4, 24, 29]. Lymphatic collectors gather initial lymphatic fluid and propel lymph forward by spontaneous contractions of the surrounding muscle layers [30]. This driving force promotes the unidirectional flow of lymph fluid into the afferent lymphatic vessels of lymph nodes [1, 31]. The afferent lymphatic vessels convey lymph into the sub-capsular sinus and along the lymph node sinus toward the efferent lymphatic vessels [1, 32]. The lymph then drains into the thoracic duct or the right lymphatic duct, and returns to venous circulation through left and right subclavian veins, respectively [1, 33, 34] (Figure 1A).

### Aging-associated changes in collector lymphatic muscle cells investiture

The primary function of collector lymphatic vessels are to transport lymph back into the blood circulatory system [2]. The intrinsic contractile activities generated by lymphatic muscle cells determine the forward movement of lymph against an adverse pressure gradient [26, 27]. The lymphangion, the structural unit of lymphatic collectors, is divided into three parts: pre-valve zone, valve zone, and post-valve zone [35, 36]. Independent contraction of lymphangions propagates the peristalsis-like wave [37].

Studies on aged lymphatic vessels have demonstrated that the aging process changes lymphatic muscle cell composition [10]. As shown in images of mesenteric lymphatic vessels (MLV) immunohistochemically labeled for actin, zones located upstream (pre-valve zones) and above (valve zones) lymphatic valves exhibit significantly less muscle cell investiture with discontinuous and irregular muscle cell organization in aged groups [10]. These low muscle cell investiture zones consist of longitudinally-oriented muscle cells which connect adjacent lymphangions [10]. Muscle cells in these zones may have an impact on lymphatic valve gating and electrical coupling between lymphangions, while aging associated changes in longitudinally oriented muscle cells may alter these two functions [10, 38, 39]. In the elderly, decreased number of muscle cells surrounding lymphatic valve may limit the ability of these cells to mediate bio-directional propagation of contractile waves [10, 38]. In addition, loss of muscle cells may lead to decrease in lymphatic productivity (mainly through the reduction of contractile frequency), impaired lymphatic valve closure and subsequent reflux of lymph in aged lymphatic collector vessels [39]. Compromised pathogen transport by aged lymphatic collectors has been shown [6], and pathogens may spread in the opposite direction of normal lymph flow due to possible disruption of lymphatic valve gating [10]. Furthermore, the thin-walled low muscle cell investiture zones in aged lymphatic vessels may transform into aneurysm-like formations at high pressure [10]. The aneurysm-like formations are the ideal places for the development of low-velocity turbulent lymph flow, and the accumulation of various molecules, pathogens, and cancer cells [10]. These noxious substances may disseminate across the thin lymphatic wall, and decrease the ability of immune system to control infectious in aging. Further experimental work are needed to confirm these perspectives.

On the contrary, the downstream (post-valve zones) lymphatic valves surrounded by circularly-oriented muscle cells do not show any significant aging-associated difference in muscle cell investiture [10]. Muscle cells in these zones constitute 92–95% percent of total vessel length with a relatively consistent muscle investiture even in aged groups [10]. As the major cells to generate the contractile force, muscle cells in post-valve zones are necessary for lymph pump activity [40]. Since the high muscle cell investiture of post-valve zones was not affected by aging, the aging-associated inhibition of amplitude of lymphatic contractility is not as prominent as the aging-associated reduction of lymphatic contractile frequency under resting condition [41, 42].

The aging process reduces the levels of proteins that regulate muscle contraction [6]. Proteomic profiling of rat mesenteric lymphatic vessels was performed on 9-month-old (adult) and 24-month-old (aged) rats [6]. The muscle contractile proteins (troponin, and myosin), cytoskeleton-associated proteins (actin, gelsolin, and dynein), and myosin binding proteins are substantially reduced in the lymphatic collectors isolated from aged rats [6]. Na+, K+, and Ca++ channels, which are involved in generation of muscle cell action potential and induction of cell depolarization, are also decreased in lymph collectors of 24-month-old rats [6]. Down-regulation of muscle contraction proteins may mediate aging-inhibited lymphatic pump activity.

### Aging-associated alteration of NO–dependent regulatory mechanisms

NO-dependent regulatory mechanisms control lymphatic contractility and lymph flow in lymphatic vessels [42]. Under normal conditions, there are multiple sources of nitric oxide (NO) in the lymphatic vasculature [26, 43–46]: 1) endothelial NO synthase (eNOS) from lymphatic endothelial cells; 2) inducible NO synthase (iNOS) from immune cells or lymphatic muscle cells; and 3) neuronal NO synthase (nNOS) from the perivascular lymphatic nerves. The role of nNOS in regulating lymphatic contractions still requires further exploration. The following section focuses on NO production from eNOS and iNOS.

eNOS in lymphatic endothelial cells is required for maintaining normal contractile events under physiological conditions [46]. During the contraction cycle, the intrinsic spontaneous pumping activities promote sustained forward flow which change pulsatile shear stress [47]. The lymphatic endothelium is highly sensitive to flow/stress and potentially generates NO [26]. The phasic generation of NO acts on lymphatic muscle layers concomitantly with the reduction of contractile frequency and tone [30, 48]. This spontaneous transient suppression of pump events is essential for increased diastolic filling of lympangions [49]. NO inhibits vasomotion primarily through the NO-induced production of cyclic GMP (cGMP) and the subsequent activation of both cGMP- and cAMP-dependent protein kinases (PKG and PKA) [49, 50]. The NO/cGMP regulatory pathway inhibits Ca++ release from intramyocellular stores and affects the pacemaker events of lymphatic muscle cells, leading to a decrease in contractile amplitude and frequency [49, 51, 52]. Gasheva et al compared the NO-dependent self-regulatory mechanism between an adult group and an aged group in the thoracic duct (TD) [13]. In adult rats, NO is produced from eNOS activity in the lymphatic endothelial cells in response to imposed flow [45], (Figure 2A). With an increase in imposed flow, the enhanced eNOS activity mediates the inhibition of the lymph pump in adult rats [48]. This inhibition reduces lymphatic pacemaker activity and contraction frequency [13]. This kind of spontaneous transient depolarization is essential for increased diastolic filling and the subsequent production of a larger contraction amplitude [45]. In contrast, the TD segment in old rats behaves differently in response to the imposed flow [13] (Figure 2B). No significant inhibition of lymph pump occurs in the aged group at high levels of imposed flow [13]. Furthermore, the contraction frequency and fractional lymph flow is unchanged in comparison with the adult group [13]. This aging-related alteration illustrates that the self-regulatory adjustment of lymphatic vessels is reduced to the changes in lymph flow [45]. Further experiments demonstrated that the reversal of eNOS/iNOS activity causes contractile functional impairment in the aged group [13].

**Figure 2:** **NO–dependent regulatory mechanisms in aged lymphatic vessels.** (**A**) In adult lymphatic vessels, the enhanced eNOS activity mediates the transient inhibition of contraction frequency to adapt the load by the increase of imposed flow. (**B**) In aged lymphatic vessels, increased iNOS level renders the contractile parameters unchanged in response to increased imposed flow.

A chronic inflammatory environment often exists in the elderly [53, 54]. Excessive NO produced by CD45+CD11b+Gr-1+ myeloid cells overwhelms the spatial and temporal NO gradients produced by eNOS during inflammation [13, 43]. iNOS- derived NO may cause continuous relaxation of peri-lymphatic smooth muscle cells (SMCs), increase of vessel diameter, and decrease of inotropy, leading to reduction of contraction strength [43]. Therefore, we proposed that increased iNOS activity in the aged causes lymphatic vessels to be less responsive to imposed flow due to the presence of chronic inflammatory environments. In addition, NO is synthesized from L-arginine as a substrate for NO synthases, particularly for eNOS [55]. Ageing-induced up-regulation of arginase, the enzyme that degrades L-arginine, reduces L-arginine available for eNOS [56]. Thus, synthesis of NO is compromised in the circulation of the elderly [57]. Decreased eNOS activity leads to the loss of ability to regulate imposed flow, and consequently, the lymphatic vessels of aged rats are unable to adapt their pumping ability to transport the increasing level of lymph flow [13, 45]. Quantitative analyses also found an aging-related reversal in eNOS/iNOS expression in the TD segment [13]. The data showed a significant decrease in the relative levels of eNOS and a dramatic increase in the iNOS levels in old rats [13]. Lower sensitivity to the imposed flow induced by iNOS causes difficulties in the maintenance of the lymphatic contraction efficiency and adequate diastolic filling [11, 13]. Therefore, the lymphatic vessels of aged rats fail to appropriately adapt their contractility to various preload/ after load challenges.

### Aging-related alteration of glycocalyx and intercellular junctions of lymphatic vessels

The lymphatic endothelial cell surface is covered by the glycocalyx layer on the lumen side [6]. The main components of the substrate layer bind to the endothelial membrane through several “backbone” molecules [58]. These molecules contain proteoglycans with a core protein and one or more long-branched glycosaminoglycan side-chains, as well as glycoproteins with short-branched carbohydrate side-chains [58–60]. Embedded in and on top of the grids of proteoglycans and glycoproteins are soluble components from blood stream [58, 61], which are also the components of lymph fluid. The glycocalyx functions as a barrier between lymphatic fluid and the endothelium to prevent immune cells and pathogens from adhering to the endothelium [6, 62, 63]. Zolla et al reported a significant loss of glycocalyx with a reduction in thickness and destruction in continuity in lymphatic endothelial membranes from aged rat [6]. This observation was in contrast with the intact, continuous layer covering cell membranes from adult lymphatic vessels [6, 18] (Figure 3A). The global proteomic analysis of ultrastructural changes of glycocalyx composition also demonstrated a dramatic difference between the adult and aged groups [6]. The thin glycocalyx layer is impaired in its ability to limit certain pathogens from adhering to the endothelial cell membrane and becomes hyperpermeable in the lymphatic vessels from aged rats [62, 64]. Thus in aged lymphatic vessels, pathogens could escape more easily from the collectors into surrounding tissue, along with an increased leakage of lymph fluid and immune cells [6, 65].

**Figure 3:** **Glycocalyx layer and intercellular junctions of lymphatic vessels during the aging process.** (**A**) In adult lymphatic vessels, the intact, continuous glycocalyx layer covers lymphatic endothelial cells. Detailed view in the box shows the normal glycocalyx layer and intercellular junctions. (**B**) Aged lymphatic vessels display thin, discontinuous glycocalyx layer. Detailed view in the box shows a significant loss of glycocalyx and adherens/tight junctions. Increased pro-apoptotic factor bak activates caspase-3 to disrupt the downstream protein β-catenin, which leads to decreased adherens junctions and impaired barrier function.

The effect of aging-related hyperpermeability is also observed in blood vessels. Adherens junctions consisting of vascular endothelial cadherin (VE-cadherin) and β-catenin maintain intercellular permeability in both blood vessels and lymphatic vessels [16, 17, 66]. VE-cadherin is a type of trans-membrane protein which connects adjacent endothelial cells through calcium-dependent homophilic binding of its extracellular domain [67]. Another component, β-catenin, is an intracellular protein that links cadherin with the actin cytoskeleton [16]. Studies have found that aging process may affect all of the adherens junctional proteins [68]. First, global proteomic profiling of the lymphatic vessels from aged rats revealed a significant decrease in cadherins [6]. The downregulation of cadherins expression results in a decreased number of adherens junction complexes [18, 69]. In contrast, β-catenin is a key regulator of barrier integrity and a known substrate for caspase 3, which is an effector caspase in the apoptotic signaling pathway [70–73]. Recent research found that increased activity of the intrinsic apoptotic signaling pathway in aged vessels leads to high expression of proapoptotic members (Bak, Bax) [18]. Caspase 3 is activated by Bak and mediates barrier dysfunction through the disruption of β-catenin [16, 18]. This series of reactions eventually causes dissociation of the VE-cadherin/ β-catenin complex and results in vascular hyperpermeability [18, 74] (Figure 3B). In addition to adherens junctions, tight junctions are an equally important determinant of vascular permeability of blood vessels and lymphatic vessels [68]. As part of the tight junction, occludin and claudin-5 showed significantly low expression level in senescent endothelial cells [68, 75]. In recent studies, cytosolic phospholipase A2α (cPLA2α), regarded as a critical protein in the formation and maintenance of tight junctions, also exhibited reduced expression levels in senescent endothelial cells [68, 76]. We hypothesize that the mechanism of intercellular hyperpermeability caused by the disruption of endothelial cell-cell junctions in aged blood vessels may also exist in aged lymphatic collectors. Further investigations are needed to delineate the detailed mechanisms related to impaired barrier function in aged lymphatic vessels.

### Aging-related changes in the composition and functionality of mast cells

Located in tissues adjacent to lymphatic vessels, mast cells produce, store and release numerous vasoactive mediators [15, 77, 78]. The vasoactive molecules serve as initiators of the immune response [78]. By releasing various inflammatory molecules, sensitized mast cells recruit certain types of immune cells to counteract the acute invasion of foreign pathogens and allergens [79]. Histamine, as the major mast cell-derived substance, is necessary to activate nuclear factor-κB (NF-κB) [80, 81]. Proper function of the mast cell/histamine/ NF-κB axis is crucial for the reactions of lymphatic vessels to pro-inflammatory stimuli [82, 83]. However, the aging process modifies the normal status of mast cells and alters the response to acute inflammation [82]. Further studies revealed that under resting conditions a higher degree of pre-activation of mast cells is located close to MLVs in aged groups [82], (Figure 4A). In basal conditions, the number of activated mast cell in all mesenteric segments is significantly higher in 24-month-old rats compared with 9-month-old rats [15, 82] (Figure 4B). Substantial inflammatory mediators, such as histamine, are released due to increased pre-activation of mast cell degranulation [15, 82]. Subsequently, activated mast cells and histamine release stimulate NF-κB signaling, which increases the production of cytokines in lymphatic tissues from aged rats [82, 84]. Eventually, high basal concentrations of cytokines and massive inflammatory factors indicate aging-associated chronic inflammatory environment [54]. Pro-inflammatory cytokines and LPS induces lymphatic endothelial cell monolayer barrier dysfunction and hyperpermeability [85]. In addition, the high osmotic pressure in aged lymphatic tissue caused by inflammatory cytokines, may contribute to the formation of lymphedema, but it remains to be proven by additional experimental work.

**Figure 4:** **Mast cells in peri-lymphatic tissues.** (**A**) Lower level pre-activation of mast cells in adult peri-lymphatic tissues under resting conditions. (**B**) In aged peri-lymphatic tissues, increased number of mast cells are activated and secret massive amounts of histamine, leading to hyperpermeability of lymphatic vessels.

An *in vivo* model of lipopolysaccharide (LPS) induced acute peritoneal inflammation of adult (9-month-old) and aged (24-month-old) rats showed that the mean number of activated mast cells increases in both age groups [82]. However, the changes between untreated and LPS-treated groups are much less in aged rats [15, 82], signifying the decreased reactivity of mesenteric mast cells to acute inflammation [82]. Activated mast cells in peri-lymphatic tissue from aged rats under basal conditions may limit the availability of sufficient numbers of mast cells for acute stimulation [15]. Consequently, no significant increase of histamine/NF-κB activation is observed in aged mesenteric tissue in response to acute inflammation [82]. The compromised mast cell/histamine/ NF-κB activation in the elderly diminishes the sensitization of CD11b positive cells, and decreases the release of NF-κB-regulated cytokines [82, 86]. Given that the CD11b positive cells could be macrophages, monocytes, and active neutrophils [87, 88], the alteration of the functional status of mast cells eventually decreases the recruitment, proper trafficking, and the activation of immune cells in aged mesenteric tissue [89]. Taken together, mast cells showed higher basal activation under resting conditions and a reduced response to acute inflammatory stimuli, which contributes to the aging-associated decrease in immune response and increase in susceptibility to infection [15, 90].

## CONCLUSIONS

In this review, we summarize the anatomical and functional changes in aged lymphatic vessels. The aging-associated remodeling of the vascular wall is characterized by decreased muscle cells and enlarged lymphatic diameter, which lead to contractile dysfunction. In addition, eNOS/iNOS disturbances diminish contractile ability with increased extrinsic lymph flow. Aging-related hyperpermeability, resulting from decreased glycocalyx and intercellular junctions, contributes to bacterial escape in aged lymphatic vasculature. Meanwhile, aging induces the basal activation of peri-lymphatic mast cells, restricting the recruitment of immune cells and affecting the reactions to acute inflammation. Thus, aging is a major risk factor for decreased pump activity, increased permeability, and delayed immune response in lymphatic system. Understanding the mechanisms underlying lymphatic aging is crucial for the treatment of vascular diseases in the elderly.
